# Electronic User Authentication Key for Access to HMI/SCADA via Unsecured Internet Networks

**DOI:** 10.1155/2022/5866922

**Published:** 2022-04-13

**Authors:** Amer Tahseen Abu-Jassar, Hani Attar, Vladyslav Yevsieiev, Ayman Amer, Nataliia Demska, Ashish Kr. Luhach, Vyacheslav Lyashenko

**Affiliations:** ^1^Faculty of Computer Science and Information Technology, Ajloun National University, Ajloun, Jordan; ^2^Faculty of Engineering, Department of Energy Engineering, Zarqa University, Zarqa, Jordan; ^3^Department of Computer-Integrated Technologies, Automation and Mechatronics, Kharkiv National University of Radio Electronics, Kharkiv, Ukraine; ^4^The PNG University of Technology, Lae, Papua New Guinea; ^5^Department of Media Systems and Technology, Kharkiv National University of Radio Electronics, Kharkiv, Ukraine

## Abstract

This paper discusses the development of new hardware and software for protecting access to HMI/SCADA systems via Unprotected Internet Networks (UPN), mainly when working remotely with confidential information. Based on the analysis carried out, it is shown that the existing vulnerabilities can be exploited by cybercriminals to steal passwords and user authentication logins. Modern protection technologies based on the OTP method have been investigated. Moreover, a new concept of information security for user authentication in UPNs when working with information remotely is proposed. The structure of the electronic key and the connection diagram based on the selected hardware modules have been developed. In addition, the two-level user identification algorithms and the firmware program code for the ATmega32U4 microcontroller are considered. Finally, to show the reliability and stability of the of the developed electronic user authentication key against any unexpected software hacking, a number of experiments have been performed.

## 1. Introduction

Industry 4.0 is a new vision in production associated with the introduction of modern digital technologies, such as Industrial Internet of Things (IIoT), Machine-to-Machine (M2M), Operation 4.0 (Ops 4.0), Big Data (BD), Cloud Computing (CC), and integration of Robotic Process Automation (RPA) with Artificial Intelligence (AI) [1]; these technologies facilitate the achieving of implementing new models for managing the production processes. One of the current ideas about modern production has found its reflection in the concept of Smart Manufacturing (SM). SM is a production concept that implements computer integration, and a high level of adaptability and a rapid change in production levels, which depends on the demand and the required tasks to solve [2]. Moreover, [2] showed that for the usage of digital information techniques that can be implemented for more flexible multiscale dynamic production systems, a single end-to-end industrial network based on IIoT is required. Indeed, the single end-to-end industrial network provides the access to the global Internet network, which supports the connection to all information control actions, besides the interaction with all constituent elements of the SM. However, implementing end-to-end systems may worsen the vulnerability of the MS systems, as a result of the information loss risk and distortion that carried out by the cyberattacks from the Internet uncontrolled sources, which could cause high economic losses and even man-made disasters. Therefore, when applying the end-to-end systems, protecting production information from the cyberattacks becomes a priority; as an example, the Stuxnet worm affected the access to the information from industrial systems Simatic WinCC SCADA [3]. Another example is the Bushehr nuclear power plant in Iran, where a worm disabled a large number of uranium enrichment centrifuges controlled by the Variable-Frequency Drive (VFD). Similarly, [4] presented the theft of IIoT production files from a Korean nuclear power plant in 2014. Indeed, the examples in [3, 4] show the urgent need to protect the access to the production SCADA/HMI information from external unprotected IoT networks during far-distance work of enterprise employees.

The work of Ali Süzen indicates that a threat of cyberattack is always present as long as there is available digital data [5]; consequently, the need for high level of cyber security is increasing. Moreover, [5] conducts valuable research into the threat of the cyberattacks sources in the Industry 4.0 ecosystem, which are listed below:

- Unsecured device connections in the control system protocols.
- The lack of regular penetration tests.
- The lack of ability to effectively manage network devices, mainly by untrained personnel, resulting in the shortage of complete prevention of the cyberattacks in the Industry 4.0 ecosystem [5].

Pang et al. proposed a new two-stream structure of SM includes specifications, organizational architecture, security, user access, databases, and hardware and software requirements [6]. However, [6] indicated that the standard solutions are left for enterprise cyber security.

The authors Efe and Isik in their publications classify the types of vulnerabilities that need to be considered and resolved in an enterprise to counter cyberattacks and increase cybersecurity [7]. However, the authors consider solutions to SM cyber security issues, only on the basis of case studies, which are not specific, but generalized in nature.

Mullet et al. evaluate methodologies and technical solutions from classic countermeasures to cyberattacks to innovative ones, for example, based on decoys and digital twins [8]. As a result, the authors have given recommendations on the cyber protection of SM, which are of a general nature without a specific solution.

The proposed new methodology for the semantic expansion and improvement of cyber security models is presented in the work of Laković et al. [9], which allows quantifying the level of existing cyber security SM, through adapted methods. At the same time, the authors do not consider security issues at the SCADA/HMI, MES, and ERP levels.

In Ferencz et al.'s article, the authors conduct MS research from a security perspective, focusing on the integration of IoT devices, and propose a theoretical architecture for the integration of SOC and IoT [10].

On the other hand, Sharma introduces the vulnerabilities and defines a cyber-defense strategy for corporate and end users, who are instructed to simultaneously implement preventive protection measures [11].

Naanani and Humayun in their work carried out a detailed review of possible cyberattacks targeting each level of Industry 4.0, as well as the consequences of these attacks and the corresponding countermeasures [12]. In addition, a multilayered framework is presented that can provide end-to-end protection against cyberattacks; however, this structure has a minimum level of protection on the Application Layer, against theft of usernames and passwords using the Phishing and Social Engineering methods to access the SCADA/HMI, MES, and ERP levels [13, 14], besides the ability to cyberattack the PLC, SCADA/HMI levels, which can lead to disruption of physical production processes.

In the work of Gómez et al., the issues of PLC, SCADA/HMI protection are considered by finding anomalies in control networks [15].

Based on the analysis of [15], it can be seen that they are aimed at tracking the possibility of a cyberattack within the IIoT network, while not paying attention to the issue of protecting the username and password from theft when logging into the SCADA/HMI system. So if the username and password are stolen, the system will consider that the user is identified with certain access parameters, resulting in making the system to be insecure and vulnerable to industrial espionage and cyberattacks.

Based on the above, in order to prevent the above commented-on errors and take into account possible other errors, the proposed work in this paper is directed to the following guidelines:

- Analyzing modern methods and technologies for user authentications; taking into account the positive aspects and identifying flaws; and developing a new concept of protecting user authentication information using modern software and hardware.
- Considering the possibility of minimizing the influence of the human factor on the loss and disclosure of the username and password content and conducting researches to resist the hacking.

## 2. General Concept of Information Protection Using Electronic Keys for User Authentication

Cracking a password is one of the most common types of attacks on any information system that uses password or username-password pair authentication. The essence of the attack boils down to the seizure of the password of the user who has the right to enter the system. In this case, the following approaches can be used [16]:

- Direct search: Enumeration of all possible combinations of characters allowed in the password.
- Selection by dictionary: The method is based on the assumption that existing words of any language or their combinations are used in the password.
- Method of social engineering: Based on the assumption that the user used personal information as a password, such as the first or last name, date of birth, and so on.

The attackers' goal is to obtain the password to guarantee granting all the rights that the original user holds. At the same time, logging in under an existing account that does not arouse suspicion among system administrators and enterprise security systems.

Therefore, the reliability of the authentication using a password or a “username-password” pair is determined by the following criteria:

- Length (the number of characters that the password contains).
- Complexity (the usage of the combinations: letters, symbols, and numbers).
- Unpredictability (the usage of the publicly available data, nicknames, dates, or any information available on social networks).

The most common cracking methods of an authentication password or username-password pair are presented in Table 1.

The presented methods of cracking an authentication password or a “username-password” pair are implemented in the following software tools; some of the most common are presented in Table 2.

By analyzing the methods of cracking the password for authentication or username/password pairs, it can be seen that reusable passwords can be compromised. As a consequence, for the safety of working with industrial information via remote SCADA/HMI, it is necessary to consider alternative security methods, which are presented in Table 3.

Let's analyze alternative authentication methods from the point of view of their application for access to industrial SCADA/HMI in unsecured networks:

- Biometrics Method: in 2017, it was proved that it is possible to recreate a fingerprint pattern from photographs taken with a digital camera from a distance of three meters [36]. In 2014, the fingerprints of the Minister of Defense of Germany were shown, which recreated from official high-resolution photographs from open sources [37]. Thus, the use of biometrics methods to implement access to industrial SCADA/HMI can be considered irrelevant and easily vulnerable.
- The Single Sign-On (SSO) method is based on setting up a trust relationship between an application known as a service provider and an access control system. The software snippet assumes local installation. This allows implementing a password store, where a single username and a single password are allowed; however, they must be entered every time to access a new application or a new site. Such a system simply stores the credentials for other applications and enters them when needed. Within the framework of these studies, this method is not suitable, since access to industrial data via SCADA/HMI is carried out through a trust relationship, and they are possible only within the industrial IIoT. Therefore, this method is not suitable for the proposed work in this paper.
- The OpenID Connect method allows Internet resources to verify the identity of the user based on the authentication performed by the authorization server. For work, the RESTful API described in the specification is used. Also, OpenID Connect defines additional mechanisms for strong encryption and digital signatures. But at the same time, some researchers believe that the OpenID protocol is vulnerable to phishing attacks, when, instead of the provider, attackers direct the end user to a site with a similar design. If the user does not notice the substitution, then he enters the authentication data (login, password). As a result, attackers can present themselves to Internet resources as a given user and gain access to the information stored on these resources. Phishing attacks are also possible when a site that supports OpenID authorization is forged in order to obtain information about the user from the provider. Using the “hidden redirect” vulnerability, attackers can create the illusion for the user that the information is being requested by this site [38].
- One-Time Password (OTP) is a one-time password method valid for only one authentication session. The one-time password can also be limited to a certain period of time. The advantage of a one-time password over a static password is that the password cannot be reused [39]. However, in some cases, the use of one-time passwords increases the risk of compromising the data of the entire system, since when an attacker accesses the OTP authentication server all system components will trust this server. However, this may increase the risk of transferring one-time passwords to attackers if the token is lost. It is worth mentioning here that often in the application, in addition to a one-time password, a reusable password should be entered, but it can also be compromised in the same way as a regular password. Finally, when OTP does not function correctly, the security of the system becomes vulnerable, such as increasing the validity period of a one-time password, which increases the possibility to guess the password, which what happened at the Banks of Sweden in 2005, and Citibank (USA) in 2006, where one-time passwords were obtained as a result of phishing attack [40].

The resynchronization of OTP tokens and authentication servers in time, as a result of which, at a certain moment, the server may have several “correct” one-time passwords. Suppose, for example, that the approximate desync time is 5 minutes and the OTP changeover period is 30 seconds. In such a situation, up to 10 “correct” passwords can exist simultaneously, which increases the likelihood of unauthorized access.

## 3. The Proposed Mythology and the Hardware

Based on the analysis of alternative authentication methods presented in Table 3, this paper proposes to modify the OTP method by using new concepts of protecting the access to the production information through unprotected networks, which are as follows:

- Implementing access in such a way that the user does not know the password and identification login.
- Complicating the password and not associating it with specific dates or associative concepts of the user (i.e., automatic generation of the username and password).
- Changing of the username and the password once a week automatically or more often without notifying the user. The period of changing the username and the password depends on the required protection level of the information and the level of security of the internal IIoT networks.
- Providing information for automatic login without using the keyboard, thus avoiding the use of keyloggers and similar spyware.
- Automatically checking of the URL, which the user visits for the protection against phishing attacks.
- Implementing two-factor user authentication.
- Providing connections to the HMI, HMI/SCADA terminal via modern USB/Tape-C/OTG interfaces, and so on, considering the protection against malicious Trojan viruses transmitted via INF/Autorun.

The structural diagram and the components' selection for the implementation of the proposed electronic key to improve the user authentication through unsecured Internet networks is illustrated in Figure 1, which shows how to implement the concept of information protection during user authentications to access HMI and HMI/SCADA systems via unprotected Internet networks.

During the development of the structural diagram, an analysis was also carried out of modern interfaces that can be used to connect to PCs, laptops, tablets, mobile phones, or external and internal terminals, through which a physical connection could be applied to ensure the authentication of user access rights to the production HMI and HMI/SCADA systems [41].

The proposed work in this paper suggests implementing the most common USB (Universal Serial Bus) 1.0–3.0 interface and its compatible Type-C and OTG counterparts. Serial interface for connecting peripherals is divided into USB 1.x (average speed 12 Mb/s); USB 2.x (average speed 25–480 Mb/s); USB 3.x (average speed 2.5 Gb/s); and Type-C or USB 3.1. All listed serial interfaces are used on 98% of industrial control systems and PCs, laptops, and modern mobile phones (except for Apple corporation). To combine these serial interfaces, adapters are used, which are free for sale and which allow you to connect the developed electronic dongle even to a hardware device of Apple corporation.

As a consequence, it is necessary to use a microcontroller with built-in extended USB functions to provide universal access to all kinds of devices, resulting in the developing of the access key that consists of three main elements: a control board, based on the ATmega32U4 microcontroller [42], was chosen due to the peculiarities of its CPU architecture, inside which, on a chip, a usb <> uart converter is implemented. Thanks to this, no drivers are required when connecting to a PC. And the computer itself recognizes the Arduino Pro Micro ATmega32U4 as a Human Interface Device (HID) device, an LCD display for displaying the necessary information [43], and a push-button control unit [44]. Analyzing the modern element base and the characteristics to solve the assigned tasks, the following hardware components of the electronic key were selected, which are shown in Figure 2.

The main characteristics of the selected hardware items are taken from the Datasheet: Arduino Pro Micro (ATmega32U4) where the Micro has built-in USB communication, eliminating the need of a secondary processor, operating voltage 5 V microUSB, Flash ROM-4Kb with dimensions of 18 × 33 mm [42], and 0.91 OLED display module with I2C connection interface; the viewing angle is more than 160°; the operating voltage is 3.3-6V with dimensions of 12 *∗* 12 *∗* 38 mm [43] and Clock button model A24 with number of contacts 4, with dimensions of 12 *∗* 12 *∗* 7.3 mm [44].

Based on the selected hardware modules, the following wiring diagram has been developed, which is shown in Figure 3.

To connect the 0.91 OLED display module, the I2C connection interface is used that requires connecting the SCL c D3 and SDA c D2 connectors to the Arduino Pro Micro. This display module was chosen because of its support for the I2C interface, which allows data transmission over two connectors (SCL, SDA) and two power supplies (5V, GND), as opposed to the Serial Peripheral Bus (SPI) interface, which uses four connectors (MISO, SCK, SS, and MOSI) for data transmission and two for power supply (5 V, GND). The 5 V power supply for the display can be taken from the VCC and GND connectors on the Arduino Pro Micro and connected to the corresponding connectors on the display. Based on the proposed structural diagram, the A24 clock model buttons is connected through a common ground, to the digital connectors (D6, D7, and D8). Accordingly, the “<<” button for menu control is connected to the D6 connector, the selection confirmation button “OK” to the D7 connector, and the menu control button “>>” to the D8 connector.

To assemble an experimental dummy of the electronic authentication key, the size form factor of a USB flash drive was chosen. The placement of all hardware modules is done on a breadboard with dimensions of 30 × 40 × 20 mm (WxDxH). When designing the topology of the printed circuit board of the electronic key, the authentication was carried out using modern CAD systems EDA Altium Designer, which reduces the overall dimensions. The obtained result of assembled prototype of the proposed electronic authentication key is shown in Figure 4.

The next step is to develop an algorithm for two-factor authentication of access to SCADA/HMI. To simplify perception, the proposed algorithm was divided to several levels.

At the first level, user authentication is performed to provide the access to the main menu of the electronic key, where a 4-digit digital access pin must be entered. Depending on the security requirements and the level of user access to the production HMI or HMI/SCADA, the minimum number of attempts in the Attempt counter, can be equal to one attempt. If pin is entered incorrectly, the electronic key is blocked for in the interval of 30 seconds before the new firmware by the security administrator is created. The algorithm of the first level of the electronic key user authentication is shown in Figure 5.

The second level of user authentication is automatic, where the electronic key management menu (Main Menu) of the user offers the name of the domains needed to perform the necessary actions. In this case, the name of the domains can be any name that is convenient for the user's association. After choosing the HMI/SCADA domain name, the electronic key copies the address line in the Web browser for verification and compares it with the domain name stored in the memory of the electronic key; if they do not match, the site is considered as “fake,” and hence the work stops, and the user receives a warning about the danger. If the domain addresses are the same, then the user puts italics on the login field and clicks the “OK” button on the key. This allows the user of the electronic key not to remember the login and password for accessing Cloud Storage of the enterprise. After automatic filling of the authentication fields, the user performs the standard action to enter in the form of clicking the “Sign in” button. Further, the received data is transferred to the enterprise's Cloud Storage server, where the user's level of the access to the information is checked on the server. If the user is defined on the server, then in accordance with his priorities and permissions, the access to information is given that is displayed in the Web browser window. The algorithm of the second level of automatic user authentication is shown in Figure 6.

The next step in the development of the HMI/SCADA user authentication electronic key is the development of software for the ATmega32U4 microcontroller. To be able to understand the required software, it is necessary to analyze the existing software development environments for microcontrollers of the whole family, which considers the following development environments: AVRStudio [45], MPLAB [46], and Arduino IDE [47]. All of the above development environments, a C ++ language or a subset of it, can be implemented. However, it is worth noting that for software development in Atmel Studio, it is necessary to additionally install the Atmel Toolchain [48]. At the same time, there is no confusion when compiling software, due to the fact that for different versions of Atmel Studio two types of compiler Atmel Toolchain and WinAVR are used [49], which complicates the perception of the compilation process. Therefore, the Arduino IDE to develop the HMI/SCADA user authentication electronic key software is chosen. The selection was based on the following factors: simplicity and ease of software development, ease of library integration, support from official Arduino developers, and a Freeware license. The enlarged logic of the firmware for the electronic key in the form of an algorithm is shown in Figure 7.

At the first stage of program development, it is necessary to connect the libraries necessary and sufficient to implement the specified functions and work with hardware modules, such as 0.91 OLED display modules 128 × 32 or tact button model A24.

In the form of constants, the password of the first level of authentication of the electronic key user to implement the algorithm (Figure 5) is set, where a 4-digit numeric password from 0 to 9 is required:

  const int pas_1 = 0;
  const int pas_2 = 0;
  const int pas_3 = 0;
  const int pas_4 = 0.

In later steps, flashing electronic access keys in secure IIoT and hence generating a random new password for the first level of electronic key automatically is required, and automatically sent to the user's phone or mail, with information about the time of its validations in the system.

The pins for connecting the clock buttons is inserted into the navigation menu for controlling the electronic key of the Arduino Pro Micro, in accordance with the connection diagram (Figure 3):

  const int pin_OK = 8;
  const int pin_UP = 6;
  const int pin_DOWN = 7.

A limit on the number of HMI/SCADA access accounts used (the maximum can be 25) is created:

int max_account_number = 5;
A function that allows dividing the key's array into columns, in the record format: site—username—login—password, is created.
typedef struct {char^*∗*^ site; char^*∗*^ name; char^*∗*^ login; char^*∗*^ password;} State;
An array in accordance with the division suggested above is created.
The flags “menu” and work with Electrically Erasable Programmable Read-Only Memory EEPROM (EEPROM) is set, where EEPROM is a type of memory that allows writing and reading data from a program, while it is not possible to clear it by rebooting the electronic key. Accordingly, implementing the storage of settings that changes “from the menu” of the device, without flashing is required, as well as a counter of attempts to maintain the first level of authentication and a counter of the timer for blocking the electronic key:
int pas_ST_1 = 0, pas_ST_2 = 0, pas_ST_3 = 0, pas_ST_4 = 0, flag_menu = 60, flag_RES_DISP = 0, msecs = 300;
int pin_OK_st = 0, pin_UP_st = 0, pin_DOWN_st = 0, account_number = 0, flag_RES_ACC = 0, timer = 0;
int address_FLAG = 1, flag_EEPROM = 125, seconds = 0;
int seconds1 = 10, seconds2 = 20;
To enter the 4-digit password of the first level of user authentication of the electronic key on the OLED display, the following function is implemented.
The function of scanning tact buttons on an electronic key is implemented by the following function:
void scan_buttons(){
    pin_OK_st = digitalRead(pin_OK);
    pin_UP_st = digitalRead(pin_UP);
    pin_DOWN_st = digitalRead(pin_DOWN);
}
Using the void setup () function, the settings for the electronic authentication key is described.
The main program for the operation of the electronic key using the void loop () cyclic function is implemented.

To flash the layout of the electronic key for user authentication in HMI/SCADA, configuration of the following Arduino IDE settings is required to work with the ATmega32U4 microcontroller (Arduino Pro Micro). In the Tools menu, in the Board section, select “Arduino Micro” and specify the Com port number, as shown in Figure 8.

After the configuration, the firmware with an ATmega32U4 microcontroller (Arduino Pro Micro) is carried out. When the electronic key is turned on for the first time, the user of the electronic key must enter a 4-digit pin to enter the main menu, as shown in Figure 9(a), and the implementation of the selection menu is shown in Figure 9(b).

The developed prototype of the electronic key for user authentication in HMI/SCADA has the following characteristics:

(i) The ability to memorize up to 25 pairs “username-password,” while the user is not obliged to know the “pair” username and does not know the “password,” which avoids the leakage of the disclosure of access data to HMI/SCADA, in contrast to software protection: Google Authenticator, SafeNet Trusted Access (STA), Microsoft MFA, and GateKeeper Enterprise, which displays the token number on the smartphone display, hardware protection: RSA token, SafeNet OTP from Thales, which displays the token number on the key display, and the visual access data, which is vulnerable.
(ii) The implemented access concepts in the developed electronic key for user authentication in HMI/SCADA, in contrast to OTP technologies, avoid the desynchronization of OTP tokens and authentication servers in time; as a result of which at a certain moment, there can be several “correct” one-time passwords on the server. For example, suppose the approximate desync time is 5 minutes and the OTP changeover period is 30 seconds; in such a situation, up to 10 “correct” passwords can exist simultaneously, which increases the likelihood of unauthorized access.
(iii) Input of information about the “username-password” pair, on public devices, occurs without using data input devices (keyboards), the data is filled in automatically, and the user simply sends them for verification to the server. This solution avoids the theft of information for a username-password pair using keyloggers, which record the sequence of typing data from the keyboard.
(iv) In case of loss and theft of the user electronic key authentication in HMI/SCADA, a “rigid system” of regulations has been developed according to the following steps:
  1. The action of the key and passwords is limited in time, depending on the security requirements, the change of the “username-password” pair occurs automatically on the server without human involvement, using random symbol generators, which reduces the likelihood of accidental disclosure to zero.
  2. If the notable four-code pin is entered incorrectly at the first level, the user authentication level, the authentication key is blocked for the set time by the administrator, during this time a new “username-password” pair is automatically generated on the server, as a result of which information about access to the HMI/SCADA is deprecated. The selection of pin by the combinatorial method is 10,000 combinations; it is not possible to perform it manually and this is provided for by the key.
(v) A high degree of protection against “dumping” information is conditionally possible only in the case of the physical theft of an electronic key, and at the same time, an attacker is not very likely to receive a firmware file in a hexadecimal format, which must be disassembled.

## 4. Practical Experiments to Test the Burglary Resistance of the Proposed Key Security

We will conduct a number of studies to check the stability of the developed electronic key against theft of information in HMI/SCADA user authentication. When introducing the developed electronic key into mass use, it is possible to use a three-level protection for reading the firmware by known methods: protection against opening the case, hidden internal breakage of the leg used by the programmer for reading, and hidden on-chip removal of the leg control logic used for reading. The first level is a refractory polymer that is resistant to acids and solvents, which does not allow reaching the crystal. The second level makes it impossible to read the programmer without special expensive tools. The third level performs a function similar to the second, but at the same time on-chip restoration of the control logic on the inner layers is practically impossible, or it requires very expensive equipment. When introducing the developed electronic key into operation, the authors recommend using the unpackaged ATmega32U4 microcontroller. In the course of an attempt to hack the firmware of an electronic key, in laboratory conditions, the authors of the article were unable to remove the “firmware clone” through the AVRDUDE program [50], since the firmware is copy-protected. Therefore, a situation when attackers managed to steal an electronic key and copy a firmware file from it in ^∗^.hex format will be simulated. A hex file is a hexadecimal file containing source code, configuration information, setting information, or other data. The format is commonly used in low-level programming when developing microcontrollers. A fragment of the firmware file of the electronic key in hex format is shown in Figure 10(a) and in Figure 10(b), in an attempt to disassemble it.

As an example, an attempt to disassemble the resulting fragment is presented in Figure 10(b), using the strcpy functions (the standard library of the C programming language, for copying a null-terminated string into a given buffer) for the ARM architecture. A fragment of the resulting assembly language code is shown in Figure 11.

The presented fragment contains the command for calculating registers and the processing, and then the cycle can be observed; however, from the presented fragment, it is impossible to understand the essence of the execution of commands and the purpose, which does not allow to open and understand the authentication passwords and the purpose; as a result, this gives an opportunity to make sure that the software hacking the electronic user authentication key in HMI/SCADA is a difficult task, even if the attackers have a source file in ^*∗*^hex format, the maximum that allowed to be viewed is the firmware code.

We can also note the strengths and weaknesses of the developed approach. This is presented in Table 4, which gives a comparative description of the developed approach and existing approaches.

## 5. Conclusions

In this paper, the processes of developing authenticating user access to industrial information through unsecured Internet networks were introduced in detail. Moreover, a number of vulnerabilities for cyberattacks were identified, such as phishing and social engineering, which are based on the human factor.

The authors analyzed the proposed new method for organizing user access to industrial SCADA/HMI. The analysis based on the concept of an unknown authentication parameters. Consequently, an electronic key based on ATmega32U4 microcontroller was developed as well. All the necessary information to enter the industrial SCADA/HMI is stored inside the firmware in accordance with the company's internal cyber security regulations, which allows generating a powerful automatic passwords and user logins without involving the user's information to remove the risk of accidental transmission of the authentication parameters to a third part. Accordingly, the authors developed a structure, selected electronic components, developed a connection diagram, and assembled an experimental model of an electronic key for user authentication of industrial HMI, HMI/SCADA. On the other hand, to protect the access to the main menu of the electronic key, the authors have developed an algorithm for the first level of user authentication and an algorithm for the second level of automatic user authentication with an electronic key for accessing information in HMI/SCADA. The firmware for the ATmega32U4 microcontroller has been developed as well, which can store up to 25 logins and passwords. To testify the proposed algorithm, a number of experiments were carried out to simulate the hacking of an electronic key, which showed high stability and reliability of the stored information, compared to the same parameters without applying the proposed development. The future work is planned to be directed to apply the proposed algorithm on more complicated networks where the information is transmitted in broadcast manor, such as the networks introduced in [51–55].

The authors are confident that the method proposed in the article will protect data with high reliability from hacking by social engineering. But this requires the implementation of all the recommendations in the proposed concept. This is based on the fact that the strength of the password is due to the fact that the user does not know the access passwords, which are automatically generated and remotely recorded on the electronic key. Moreover, depending on security requirements, access passwords can be changed each time the dongle is connected to a secure device (PC, etc.) in the local network without warning the user. The authors are also confident that if the developed key is stolen, the data will be protected from hacking during the first 24 hours. This is based on the fact that during this time you can change access passwords or block an account. At the same time, the authors understand that there is a possibility of physical hacking of the prototype microcontroller. But this method of hacking requires expensive equipment. Moreover, this hacking method leads to the destruction of the key.

## Figures and Tables

**Figure 1:** Block diagram of the electronic key for user authentication in HMI/SCADA.

**Figure 2:** Hardware components of the electronic key. (a) Arduino Pro Micro (ATmega32U4) [42]; (b) 0.91 OLED display module 128 × 32 [43]; and (c) button clock model A24 [44].

**Figure 3:** Electrical connection diagram.

**Figure 4:** Assembled prototype of the electronic authentication key. (а) Top view. (b) Bottom view.

**Figure 5:** Algorithm of the first level of user authentication with an electronic key.

**Figure 6:** Algorithm of the second level of automatic user authentication with an electronic key to access information in HMI/SCADA IV. Development of the software for the functioning of the proposed electronic key.

**Figure 7:** Enlarged algorithm of the electronic key firmware operation.

**Figure 8:** Arduino IDE settings for flashing user authentication electronic key in HMI/SCADA.

**Figure 9:** Checking the functionality of the electronic user authentication key in HMI/SCADA. (a) The first level of user authentication. (b) Main menu for electronic key control.

**Figure 10:** An attempt to hack the firmware of the electronic key. (a) A fragment of the firmware in hex. (b) Disassembling the firmware fragment.

**Figure 11:** Fragment of the electronic key firmware in assembly language.

**Table 1:** Methods for cracking the authentication password or username-password pair.

Method	Description
Dictionary attack [17]	The method involves using a list of words to compare with user passwords.
Brute force attack [18]	The method uses algorithms that combine alphanumeric characters and symbols to come up with passwords for the attack. For example, a password with the value “password” can also be used like the word p @ $$ using a brute force attack.
Rainbow attack [19]	The method uses precomputed hashes (md5), a ready-made database of hashes is generated or bought, and then it is compared with the hashes to be cracked.
Guessing [20]	The method assumes guessing the most common passwords (qwerty, password, and admin). Usually used or set as default passwords. If they have not been changed or the user is careless when choosing passwords, then they can be easily compromised.
Spidering [21]	The method of social engineering. Most organizations use passwords that contain company information. This information can be found on company websites and social networks, such as Facebook, Twitter, and so on. Spidering collects information from these sources to compile word lists. The wordlist is then used to carry out dictionary and brute force attacks.

**Table 2:** Software tools for cracking authentication passwords.

Name of the tool	Description
John the Ripper [22, 23]	Uses command line to crack passwords. This makes it suitable for advanced users who are comfortable working with teams. It uses a wordlist to crack passwords. The program is free, but the wordlist is not.
Cain and Abel [24, 25]	Used for password cracking methods: dictionary attack, brute force, and cryptanalysis. Unlike John the Ripper, Cain and Abel uses a graphical user interface.
Ophcrack [25–27]	Is a cross-platform, Windows password cracker that uses rainbow tables to crack passwords. It works on Windows, Linux, and Mac OS. It also has a module for brute force attack attacks among other features.

**Table 3:** Alternative authentication methods.

Method	Description
Biometrics [28, 29]	These are unique biological and physiological characteristics that make it possible to establish a person's identity. There are five most common types of biometrics: fingerprint, facial, voice, eye iris, and palm and finger vein patterns.
Single sign-on (SSO) [30, 31]	An authentication method that allows users to securely authenticate to multiple applications and sites at once using a single set of credentials.
OpenID Connect (OIDC) [32, 33]	Describes a metadata document RFC that contains most of the information needed for any application to sign in. This includes information such as the used URLs and the location of the service signing public keys.
One-time password (OTP) [34, 35]	It is a password that is valid for only one authentication session. The one-time password can also be limited to a certain period of time. The advantage of a one-time password over a static password is that the password cannot be reused. Thus, an attacker who intercepted data from a successful authentication session cannot use the copied password to gain access to the protected information system.

**Table 4:** Comparative characteristics of the developed approach and existing approaches.

Hacking methods (software and hardware)	Authentication methods				
	Biometrics	Single sign-on (SSO)	Open ID connect (OIDC)	One-time password (OTP)	Developed approach
John the Ripper	+	−	−	−	+
Spidering	±	−	−	−	+
Cain and Abel	+	−	−	+	±
Dictionary attack	+	−	−	−	+
Brute force attack	+	−	−	−	+
Ophcrack	+	−	−	+	+
Create a clone	−	+	+	+	+

+ not vulnerable, ± partially vulnerable, and − vulnerable.

## Data Availability

The data used to support the findings of this study are included in the article.
